# Clinical management of chronic mercury intoxication secondary to skin lightening products: A proposed algorithm

**DOI:** 10.17305/bjbms.2020.4759

**Published:** 2021-06

**Authors:** Fitri Fareez Ramli

**Affiliations:** Department of Pharmacology, Faculty of Medicine, Universiti Kebangsaan Malaysia, Cheras, Kuala Lumpur, Malaysia

**Keywords:** Mercury, cosmetics, skin-lightening, skin-whitening, bleaching, nephrotic syndrome, neuropsychiatry, dementia

## Abstract

Mercury is a toxic substance that is commonly used in skin lightening products. Various effects on humans have been observed, which affect both users and non-users. Many studies reported delayed diagnosis and treatment, even after weeks of hospitalization. The possible reasons are non-specific clinical manifestation and lack of awareness and knowledge regarding chronic mercury intoxication secondary to skin lightening products. A thorough history of mercury exposure is crucial. Physical assessment and relevant supporting tests are indicated to establish a diagnosis. Blood and urine mercury levels are an essential examination for diagnosis and monitoring of the progress and response to treatment. The primary treatment is the discontinuation of the skin lightening products. Chelation therapy is not mandatory and is usually indicated for symptomatic patients. The prognosis depends on the duration of the product use, concentration of mercury in the skin product, and the severity of clinical presentation.

## INTRODUCTION

Mercury is a toxic substance that is commonly used in skin lightening products. Mercury use prevails due to its ability to produce a dramatic whitening effect, mainly when used at a very high amount. According to the World Health Organization, the mercury levels in skin lightening products should be less than one part per millions (ppm) [1]. Despite tight regulations in many countries, numerous skin lightening products contain more than thousands of the acceptable limit of mercury levels. According to the study conducted in the US, nearly half of the mercury-containing products had a very high mercury level, exceeding 10,000 ppm [2]. Skin-lightening products are manufactured in many countries, such as the UK [3], Mexico [4-8], Lebanon [9], Taiwan [9], Indonesia [10], China [2,11,12], Japan, Thailand, the Philippines, and Jamaica [2]. Both online and physical stores, such as beauty shops, stores [13] and flea markets, as well as relatives and friends [14] contribute to the availability and widespread use of skin lightening products.

Inorganic mercury used in skin lightening products has various effects on humans. Two common forms of inorganic mercury are mercurous (Hg^+^) and mercuric (Hg^2+^) salts [15]. The effects are not only limited to the users, but people who are in close contact with the user may also be affected [4,16-18]. Both the user and non-user may exhibit no symptoms or may develop mild to severe symptoms and signs. Neurological and renal impairment is the common manifestation of chronic mercury intoxication. Cardiovascular [4,19] and dermatological conditions [20] may also develop to a lesser extent. The latency of sign and symptom manifestation ranges from months to years. Also, the mercury levels in the body may not correlate with the symptoms as the abnormal levels may develop no symptoms [14].

Many case reports showed that patients with chronic mercury intoxication had visited the doctor for the symptoms associated with their current condition but that was not detected. Some of the patients with severe presentation who require hospitalization get proper chelation therapy only after 2–3 weeks from admission due to delayed detection [6,14]. The reasons for the delayed diagnosis and treatment may be 1) non-specific clinical signs and symptoms such as headache and pain, 2) clinical presentation is similar to diseases that may be caused by other etiology such as nephrotic syndrome and systemic lupus erythematous, and 3) lack of knowledge and awareness on chronic mercury intoxication. This review aims to elaborate on chronic mercury intoxication secondary to skin lightening products based on the previous case reports and studies. The elaboration includes the mechanisms, pathophysiology, clinical signs and symptoms, and management of chronic mercury intoxication. To my knowledge, there is no specific algorithm formulated for the management of this condition. The proposed algorithm aims to provide a guide for the healthcare practitioners on the management of chronic mercury intoxication secondary to skin lightening products.

## MECHANISM

Mercury competes with copper ions for tyrosinase, an enzyme involved in melanogenesis [15,21]. Binding of mercury ions causes inactivation of tyrosinase enzymes. Reduced melanin content makes the skin fairer. Mercury from skin lightening products gets into systemic circulation via penetration of the skin through the epidermis, sebaceous gland, sweat gland, and hair follicles [22]. The extent of mercury absorption depends on product formulation [23], skin integrity, and lipid solubility of the vehicle [22].

## PATHOPHYSIOLOGY

Mercury exists in three forms, namely elemental, inorganic, and organic. Most of the studies on skin lightening products reported the presence of inorganic form. This form of mercury has low lipid solubility, hence it does not readily cross the blood-brain barrier (BBB). So, how does inorganic mercury contribute to neurological symptoms and signs? Mercury ions can inhibit Na^+^-K^+^-ATPase in the cerebral cortical microvascular area [24]. The inhibition of Na^+^-K^+^-ATPase causes damage to this area because 1) the accumulation of Na^+^ ions in endothelial cells causes injury to the BBB and 2) the accumulation of K^+^ ions in the intercellular compartment induces chloride shift via K^+^-dependent cotransporter into glial cells. The accumulation of potassium and chloride ions in glial cells, such as astrocytes, increases intracellular osmotic pressure, leading to the movement of water intracellularly and resulting in swelling [25]. Morphological changes in the BBB facilitate mercury transfer into the brain [24,26]. Inorganic mercury tends to accumulate in motor parenchyma. The accumulation in this area leads to increased oxidative stress and induced cytotoxicity and apoptosis with subsequent functional loss of motor neurons and astrocytes [27].

Moreover, inorganic mercury has been shown to induce neuronal degeneration, which may manifest as early-onset dementia [9]. The mechanism of inorganic mercury effect on dementia is associated with its high affinity to selenium and selenoproteins. Selenoproteins such as selenoprotein P (SelP), thioredoxin reductase, and glutathione (GSH) peroxidase are essential as antioxidants in redox reactions and for maintaining an adequate level of GSH in the brain. Interaction of mercury with SelP leads to an increase in oxidative stress, accumulation of amyloid plaque and neurofibrillary tangles (NFT), and apoptosis. Progressive accumulation of amyloid plaque and NFT causes neuroinflammation and degeneration affecting cognitive function, short-term memory, and attention [28].

The kidney is the main organ for inorganic mercury accumulation. Membrane disruption can occur upon contact with mercury. Free mercury in the proximal convoluted tubule is rapidly taken up by the epithelial cells through pinocytosis [29]. Inorganic mercury binds to intracellular proteins with free sulfhydryl groups such as GSH. The depletion of GSH increases oxidative stress intracellularly [30], leading to cellular degeneration, apoptosis, or necrosis [29,31].

Moreover, other proteins containing sulfhydryl groups are also affected – the interaction with cytoskeleton structures such as tubulin further compromises cellular activities and structures [31]. Tubular injury is mainly observed and characterized by elevated levels of tubular markers such as β_2_ microglobulin and N-acetyl-β-D-glucosaminidase (NAG) [32]. Mercury can induce glomerulopathy secondary to immune response, characterized by an elevated level of immunoglobulin (Ig)E and production of autoantibodies. Proteinuria develops secondary to IgG deposition along the glomerular basement membrane [33].

Other than the kidney and the nervous system, exposure to inorganic mercury may cause skin lesions. Hwang et al. [34] reported that inorganic mercury is able to cause membrane cell damage as well as cell death of keratinocytes. The metallothionein protein expression is increased, protecting keratinocytes from the damaging effects of mercury [34]. The accumulation of mercury granules in the dermis causes skin hyperpigmentation due to absorption from sebaceous glands and hair follicles. Nail discoloration and brittleness may develop secondary to mercury deposition in keratin [35]. Sympathetic activation can occur as catecholamines and vanillylmandelic acid accumulate secondary to catecholamine-O-methyltransferase (COMT) inhibition. Inorganic mercury binds to the sulfhydryl group of COMT cofactor, rendering it inactive [36]. This condition is common in children but rare in adults, and the reason is poorly understood.

## DIAGNOSIS

### History

History taking is a fundamental step for the diagnosis and management of the disease. The patient’s chief complaint, as well as other associated symptoms, must be obtained. Underlying diseases, such as diabetes mellitus, hypertension and renal disease, should be sought [37]. Self-treatment history, such as the use of non-steroidal anti-inflammatory drugs and herbal medicine, may give insight to possible etiology of nephrotic syndrome. It is essential to obtain information regarding potential mercury exposure such as occupational, dietary, and domestic or the use of skin lightening products, particularly for those presented with non-specific neuropsychiatry symptoms and nephrotic syndrome. More information, such as frequency and duration, should be acquired [10]. The brand, manufacturer, country of origin, and source of the product should also be obtained.

### Signs and symptoms

Patients with chronic mercury intoxication may have no symptoms despite high levels of mercury in the body [5,14]. For those who develop symptoms, there is a wide range of symptoms that are usually non-specific and may resemble disorders or diseases such as nephrotic syndrome [3,37], systemic lupus erythematosus [3], pheochromocytoma [14,19], polyneuropathy, and dementia [9] (Table 1).

**TABLE 1:** The characteristics of cases, duration of exposure, product properties, clinical manifestation, choice of treatment and patient prognosis, or contact with mercury-containing skin lightening products

The main symptoms of chronic mercury intoxication are neurological and renal impairment. The neuropsychiatric presentations are usually not specific and may include headache [4,8,9,17,18], dizziness [4,17,18], irritability [4,8,13,18], agitation [4,19], delirium [4,6], seizures [9,19], dementia [9], fatigue [8,16], pain [9,13], blurry vision [6], vision changes [16], speech disturbance [6,9], memory loss [8,9,13,16], forgetfulness [4,17], disorientation [9], emotional liability [7], shyness [14,19], dysthymia [19], depression [4,13,17,18], anxiety [4,13,18], nervousness [8,16], worriedness [18], personality changes [18], decreased concentration [18], trouble making decision [18], sleep disturbance [4], insomnia [7,8,13], dreams [13], tremors [7,8,13,19], muscle twitching [4], weakness [4,6,8,16,18], muscular hypotension [19], paralysis [18], numbness [4,17], tingling sensation or burning sensation [4,7,8,17], gait disturbance [4,6], and refusal to walk [4]. Renal involvement is characterized by frothy urine [10] and facial [3,32] and limb edema [3,12,32,37,38].

Skin manifestation is not shared. Dermatological symptoms and signs include itchiness [7,19,20], malar rash [7], intermittent flushing [7], palm rash [19], papulovesicular lesions [20], erythema of the palms and soles [7], and hair loss [18]. Systemic allergic dermatitis or baboon syndrome is a rare dermatological manifestation in inorganic mercury intoxication but has been reported before [20].

Cardiovascular signs are rare in adults with inorganic mercury intoxication but have been reported in children [4,14,19]. Three studies reported children aged 17 months–17 years presented with prominent neurological symptoms with hypertension [4,14,19], tachycardia [4,19], and profuse sweating [4].

Other symptoms include fever [14], metallic taste [8], gingivitis [13], sore gum [16], gum bleeding [18], hypersalivation [7], sialorrhea [7], eye irritation [18], eye twitching [18], rhinorrhea [14], congestion [14], loss of appetite [4,14,19] and weight loss [19], constipation [14], and arthralgia [14]. In view of a wide range of symptoms, further investigations are essential to rule out differential diagnosis.

### Physical examination

A general examination is vital as it can give us some clues to establish a diagnosis later. It includes patient consciousness level, orientation (time, person, and place), behavior, gait, and skin complexion. Fair or light-colored facial skin complexion compared to other parts of the body may give us a clue of skin lightening product use in Asian users [3,10,37]. Vital signs measurement such as heart rate, blood pressure, respiratory rate, and temperature is essential. Hypertension and tachycardia are commonly present in children [4,14,19]. Examination of other systems such as the respiratory, cardiovascular, abdomen, and central nervous system are crucial to differentiate with other conditions but appear normal in some cases [10,37].

### Investigation

Due to non-specific features of chronic mercury intoxication, appropriate investigations must be carried out. Complete blood count, renal and liver function tests, urinalysis, and chest and abdominal radiography may be conducted to rule out other diseases associated with the symptoms. These results can be normal in some patients.

Neurological tests, such as electromyography examination, can be conducted [13]. The results may be either normal or abnormal, with characteristics of slow sensory nerve conduction velocity [13] and reduced amplitudes.

Magnetic resonance imaging (MRI) is indicated in unexplained encephalopathy and seizure [19]. The use of MRI is essential to rule out other brain pathologies associated with increased serum neuron-specific enolase levels such as neuroblastoma or small cell lung cancer [9]. Serial MRI is recommended to monitor the progression or improvement of the brain lesion after chelation therapy [9,19]. Benz et al. [19] reported no brain lesion during the initial assessment of a 4-year-old child presented with clonic seizures secondary to mercury exposure following three months’ use of skin lightening products. Hyperintense lesions in the subcortical white matter in the parieto-occipital and temporal region of the right hemisphere and the paramedian aspect of the parietal lobe developed on day 7 of chelation therapy. Worsening of neurological conditions and increased mercury urine levels were also observed. The follow-up 4 months later with brain MRI revealed complete resolution of brain lesions. In contrast, Zellner et al. [9] reported the emergence of new hyperintense brain lesions during a 3-month follow-up in a patient with dementia and epilepsy secondary to 6-year mercury exposure. Initially, the hyperintense brain lesions were seen in supratentorial regions, particularly in frontal regions and semioval center. New lesions seen were located in the subcortical region of the left temporo-occipital. However, the clinical symptoms of this patient improved despite the emergence of new lesions. This contrasting finding may be explained in terms of the duration of exposure and age. Longer duration and older age are the potential for a slow, more reduced response.

An electroencephalogram (EEG) is indicated for the patient presented with seizures. Benz et al. [19] reported abnormal slow generalized (5–6/s) wave in a 4-year child presented with seizure. In contrast, Zellner et al. [9] reported no abnormality in EEG of a patient with chronic mercury intoxication with epilepsy and dementia.

The instrument for psychiatry assessment, such as Hamilton Depression Scale-17 (HAMD-17), can be utilized for patients presented with psychiatry symptoms. Sun et al. [13] reported that all 16 Chinese patients presented with various neuropsychiatry symptoms had abnormal values of HAMD-17.

Proteinuria [10,12,13,18,32,37,38] is one of the most common positive findings in patients with renal involvement. Some patients developed signs of nephrotic syndrome, which include hypoalbuminemia [37,38], hypercholesterolemia [37] and proteinuria [37], with a clinical presentation of edema [37]. Other tests to exclude the potential cause of nephrotic syndrome such as antinuclear antibodies [10,32,37], anti-deoxyribonucleic acid (DNA) antibody [32], anti-double-stranded DNA antibody [32,37], anti-neutrophil cytoplasmic antibody [10,37], streptococcuwwws hemolysin O antibodies [32], anti-glomerular basement membrane antibody [32], serum complement [10,37], anti-hemorrhagic fever virus antibody [32], hepatitis B [3,10], and hepatitis C [3,10] are usually negative. Renal biopsy revealed minimal changes disease mainly in patients with short duration of exposure, between 2 and 11 months [12,32,37]. Glomerular findings range from normal [12,32] to minimal abnormality [10]. Other changes include the granular deposition of immunoglobulins and complements in mesangium [12], capillary wall [10], and subepithelial region [10]. The diffusion of the podocyte foot processes is another common finding [12,32]. Other studies reported membranous nephropathy [3,10]. The distinct features of membranous glomerulopathy are the thickening of the basement membrane and subepithelial dense deposits [3,38].

Measurement of endocrine parameters such as thyroid function test and catecholamine levels is essential in the case of weight loss with hypertension [14,19]. Elevation of catecholamines such as epinephrine, norepinephrine, and dopamine is common in children with those conditions [14,19]. Imaging is necessary to rule out pheochromocytoma, the differential diagnosis with weight loss, hypertension, and elevated catecholamines. The absence of adrenal mass on ultrasound and MRI abdomen rule out pheochromocytoma [14,19].

Mercury levels are required to determine the need for chelating therapy and monitoring the effect of the treatment. The levels can be obtained using hair, blood, and urine. Hair is used for the measurement of mercury level because of mercury ability to bind to sulfhydryl groups of keratin in hair. However, the use of hair is only limited to organic mercury cases as it is readily accumulated in hair and has a high correlation with organic mercury in blood [39]. The use of hair in inorganic mercury intoxication assessment is limited due to 1) possible exogenous contamination, 2) pre-analysis preparation requirement, 3) inorganic mercury mainly accumulates in the kidney, and 4) a wide range of normal values [39]. Urine mercury is more suitable to assess inorganic mercury levels as the kidney is the main organ for its accumulation [39]. Both random and 24-hour urine samples can be used to measure urine mercury levels.

The measurement of mercury levels in skin lightening products is essential to find an association between mercury levels in the body and patient clinical presentation. Disproportionate clinical manifestation and mercury levels may indicate the presence of other elements that may contribute to a more severe presentation. Mudan et al. [6] reported the presence of organic mercury elements in skin lightening products used by a patient presented with severe neurological symptoms. In this case, the initial analysis found relatively low mercury content in the product compared to mercury levels in the body. Measurement of other forms, such as organic mercury levels, is essential in the case of disproportionate clinical manifestation. Most of the studies on chronic symptomatic cases reported the use of skin lightening products with mercury levels exceeding 1000 ppm [3,4,6-10,12,14,16-19,37,38]. However, mercury levels as low as 6.8 ppm have been reported to produce symptoms with longer duration [32].

## MANAGEMENT

The mainstay treatment of chronic mercury intoxication is the removal of mercury-containing products (Figure 1). Discontinuation alone may contribute to a spontaneous reduction in blood and urine mercury and improvement of the symptoms [11,17,18]. Supportive management is essential to maintain the airway, breathing, circulation, and nutrition of the patient [6].

**FIGURE 1:** Algorithm: Clinical management of chronic mercury intoxication secondary to skin lightening products.

Chelation therapy may be considered in certain conditions, such as in the case of 1) symptomatic patients with abnormal urine mercury levels or 2) patients with 24-urine mercury >100 μg/L with a two-fold increase in urine mercury upon challenge test with dimercaptosuccinic acid (DMSA) [18]. Chelation therapy aims to form a stable complex between the chelator and mercury to facilitate mercury excretion [40,41]. DMSA [6,9,18] and D-penicillamine (DPA) [7,12,37] are chelating agents of choice for chronic mercury intoxication. Dimercapto-1-propanesulfonic acid (DMPS) is used in limited cases but is useful as an alternative in the case of an adverse event of DMSA [9]. The response to chelation therapy ranges from complete resolution to inadequate response. Sun et al. [13] reported complete resolution of proteinuria, pain, anxiety, and depression after 3 to 5 chelation courses within 4–8 weeks among 16 Chinese women. This study population had 4–13 weeks of latency before the onset of symptoms. However, chelation therapy should not be used as a universal treatment in chronic mercury intoxication as harmful adverse reaction may occur due to reactivation of toxic metals and removal of essential elements because chelators are not metal-specific [42,43]. Furthermore, the precise and latent effects due to chelation therapy are not yet established [42]. The clinical benefit of chelating agents is uncertain according to some studies [42,44]. Proper assessments in terms of sources of mercury exposure, symptoms and signs, lab investigations, and risks and benefits of chelation are crucial before the commencement of chelation therapy [42,43].

In nephrotic syndrome secondary to mercury intoxication, chelation therapy (DPA, DMPS) alone or in combination with other treatments, such as steroids and diuretics, has been shown to have a good prognosis with complete resolution of signs, symptoms, and lab parameters [12,32,37]. Normalization of urine mercury levels takes longer than the blood levels within the ranges of 6–16 months [12,32] and 1–7 months [12,32], respectively. Both duration of use and mercury levels in skin lightening products determine the latency of clinical manifestation.

However, chelation therapy may worsen patient condition temporarily and with dramatic improvement later [19]. Worsening of the symptoms may be partly due to the redistribution of inorganic mercury from the kidney and liver to motor axons following treatment with DMSA [19,45] or DMPS [45].

In contrast, other studies reported inadequate response to treatment. Mudan et al. [6] reported rapid deterioration of neurological symptoms in 47-year-old Hispanic-American patients within 2 weeks from the initial presentation and who required hospitalization. Further investigation found elevated blood and urine mercury with levels of approximately 1500 times and more than 120 times the reference values, respectively. Surprisingly, they also detected elevated blood methylmercury levels, an ingredient that is not commonly found in skin whitening products. The poor improvement despite prolonged chelation therapy with DMSA may be due to the presence of a toxic level of methylmercury [6]. Ori et al. [14] reported a 17-month girl who was exposed to a mercury-containing product with a level of 27,000 ppm for 4–5 months. The exposure of mercury via inhalation of mercury vapor, close skin-to-skin contact with her mother and grandmother, skin-to-contaminated household items, and incidental ingestion of mercury attached to a contaminated surface may have contributed to mercury intoxication. This patient received chelation therapy DMSA for more than a month. Although the patient had improved condition, the residual neurological deficit was still noted during follow-up at 7 months from admission [14].

Decontamination of household items and air is required to eliminate the source of mercury and prevent recurrence of the symptoms and signs of mercury intoxication. Removal of the products is compulsory, as this is the primary source of mercury. Moreover, assessment of the household items and air quality is required to determine further action. Ventilation and heating can improve indoor mercury levels. Garden sulfur powder is useful for the decontamination of household items, personal items, as well as the body part with high mercury levels. Disposal of the items with high levels of contamination is necessary to reduce mercury levels immediately [4,17]. In the case of a high level of contamination (mercury levels >10,000 ng/m^3^), temporary occupancy exclusion of the house is recommended [14].

## CONCLUSION

Chronic mercury intoxication may cause a wide range of symptoms and signs that are not specific and resemble diseases with other common causes. Taking proper and thorough history regarding mercury exposure through skin lightening product use, dietary, domestic, or occupational factors is essential. This can guide the doctor to investigate further, remove the cause of the disease, and start the treatment immediately. Early detection has been shown to produce good prognosis. Awareness and knowledge regarding chronic mercury intoxication secondary to skin lightening products are crucial as the products are widely available.
